The article "Related Factors of Cerebral Hemorrhage after Cerebral Infarction and the Effect of Atorvastatin Combined with Intensive Nursing Care" was retracted in 2023. Reasons: signs of a paper mill; compromised peer review; unreliable results or conclusions.

# Related Factors of Cerebral Hemorrhage after Cerebral Infarction and the Effect of Atorvastatin Combined with Intensive Nursing Care

**DOI:** 10.1155/2022/9546006

**Published:** 2022-07-31

**Authors:** Qian Yang, Yuedong Yang, Xiaoting Li

**Affiliations:** ^1^Internal Medicine Department, Leshan Vocational and Technical College, Leshan City Sichuan Province, China; ^2^Neurology Department, The People's Hospital of Wutongqiao District, Leshan City, 614000 Sichuan Province, China

## Abstract

**Background:**

Cerebral infarction is a common neurological disease with high incidence, which is the main factor causing death and disability in adults in China. Cerebral hemorrhage transformation is a common clinical complication. High NIHSS score at admission, atrial fibrillation, and small artery occlusion cerebral infarction can increase the risk of cerebral infarction complicated with hemorrhage transformation.

**Aim:**

To explore the related factors of cerebral hemorrhage transformation after cerebral infarction and the value of atorvastatin calcium tablets combined with early intensive care measures.

**Methods:**

In this study, a case-control study was conducted. Sixty patients with hemorrhagic transformation after cerebral infarction admitted to the Department of Neurology of our hospital from January 2017 to June 2021 were selected as the observation group, and 90 patients with cerebral infarction without hemorrhagic transformation during the same period were selected as the control group. The risk factors of hemorrhagic transformation after cerebral infarction were analyzed.

**Results:**

The results of logistic regression model showed that the increased National Institutes of Health Stroke Scale (NIHSS) score at admission, hypertension, atrial fibrillation, TOAST classification of small artery occlusion, and large infarction lesions were the risk factors for hemorrhagic transformation in patients with cerebral infarction (*P* < 0.05). After 2 weeks and 4 weeks of treatment, the NIHSS scores of the intervention group were lower than those of the conventional group (*P* < 0.05). NIHSS scores of the two groups after treatment were significantly lower than those before treatment (*P* < 0.05). After three months of treatment, the patients in the intervention group with GOS score of 5 points accounted for 16.67%, and the patients with GOS score of 4 points accounted for 56.67%. The patients in the conventional group with GOS score of 5 points accounted for 6.67%, and the patients with GOS score of 4 points accounted for 33.33%. The prognosis of the intervention group was better than that of the conventional group on the whole (*P* < 0.05).

**Conclusion:**

Patients with hypertension, large infarction lesions, high NIHSS score at admission, atrial fibrillation, and small artery occlusion cerebral infarction can increase the risk of bleeding transformation in patients with cerebral infarction. For patients with bleeding transformation, atorvastatin calcium tablets combined with early intensive nursing intervention has a certain value for improving the prognosis of patients.

The article "Related Factors of Cerebral Hemorrhage after Cerebral Infarction and the Effect of Atorvastatin Combined with Intensive Nursing Care" was retracted in 2023. Reasons: signs of a paper mill; compromised peer review; unreliable results or conclusions.

## 1. Introduction

Cerebral hemorrhage transformation is one of the common complications in patients with acute cerebral infarction, which can lead to the complication of the disease, affect the application of anticoagulant or antiplatelet drugs, cause the interruption or delay of the treatment plan, and give rise to treatment failure. It is a risk factor for the prognosis of patients with acute cerebral infarction [1, 2]. Once cerebral hemorrhage transformation occurs, antiplatelet drugs and anticoagulant drugs should be discontinued immediately, and symptomatic treatment such as dehydration, brain protection, nerve nutrition, and improvement of brain metabolism should be given appropriately to prevent secondary brain injury. But there are still quite a few patients with poor efficacy and poor prognosis [3, 4].

Basic research suggests that too high levels of low-density lipoprotein cholesterol and total cholesterol can lead to changes in vascular permeability, local inflammatory response, and lipid peroxidation, which can increase the risk of vascular rupture [5, 6]. Therefore, whether lipid-lowering therapy can reduce cerebral hemorrhage in the treatment of cerebral hemorrhage after cerebral infarction is worthy of further study. Atorvastatin calcium tablet is a representative of statin lipid-lowering drugs. In addition to lipid-lowering effect, it also has anti-inflammatory, stable plaque, and other pharmacological effects [7, 8]. This study explored the related factors of cerebral hemorrhage transformation after cerebral infarction and the value of atorvastatin calcium tablets combined with early intensive care measures, which were reported as follows.

## 2. Materials and Methods

### 2.1. General Information

60 patients with hemorrhagic transformation after cerebral infarction admitted to the Department of Neurology of our hospital from January 2017 to June 2021 were selected as the observation group, and 90 patients with cerebral infarction without hemorrhagic transformation during the same period were selected as the control group.

Inclusion criteria are as follows: (1) the age of the subjects ranged from 19 to 79 years. (2) The diagnostic criteria of patients with cerebral infarction refer to the criteria in the “Guidelines for Diagnosis and Cure of Acute Ischemic Stroke in China 2014” [9]. (3) The diagnostic criteria of patients with cerebral hemorrhage refer to the criteria in the “Guidelines for Diagnosis and Cure of Cerebral Hemorrhage in China (2014)” [10]. (4) Patients were admitted to the hospital within 24 hours after cerebral infarction and confirmed by CT and MRI. (5) All patients were treated in the department of neurology in our hospital, and no transfer treatment occurred. (6) The research programme meets the requirements of the medical ethics expert group of our hospital by signing informed consent with their families. Exclusion criteria are as follows: (1) intracranial space-occupying lesions; (2) patients with history of craniocerebral trauma; (3) coagulation dysfunction disease; (4) intracranial infectious diseases; (5) dementia, psychosis, and typical medical history; (6) having contraindications for anticoagulation and thrombolysis; and (7) patients with coronary stent implantation, cardiac bypass grafting, and severe heart failure in recent 2 months.

The article "Related Factors of Cerebral Hemorrhage after Cerebral Infarction and the Effect of Atorvastatin Combined with Intensive Nursing Care" was retracted in 2023. Reasons: signs of a paper mill; compromised peer review; unreliable results or conclusions.

### 2.2. Treatment Measures

Both groups were given basic treatment. In the early stage of cerebral infarction, rt-PA thrombolytic therapy, aspirin antiplatelet therapy, low molecular weight heparin anticoagulant therapy, angiotensin converting enzyme inhibitor antihypertensive therapy, and insulin hypoglycemic therapy were given to patients with hyperglycemia. Once cerebral hemorrhage conversion was found, thrombolytic therapy, antiplatelet therapy, and anticoagulant therapy were discontinued. Oral atorvastatin calcium tablets (Fujian Dongrui Pharmaceutical Co., Ltd.) 40 mg, once a day, were taken before bedtime.

### 2.3. Nursing Measures

The conventional group was given routine nursing measures at the same time. The patients kept absolute bed rest, given oxygen inhalation, closely monitored the vital signs of the patients, avoided adverse sound and light stimulation, and administered on time according to the doctor' s advice. If abnormalities are found, they should be reported to the doctor in time.

Patients in the intervention group received early intensive care measures. They were absolutely bedridden for 1–2 weeks in the early stage, and the head of the bed was raised by 15–30°. When necessary, the restraint belt could be used to prevent falling from bed. Timely help patients turn over, knock back, and massage compression site, in order to prevent pulmonary infection and bedsore. Give rich nutrition, low fat, and low salt diet and drink more water, to prevent blood flow retardation. Give patients atorvastatin orally on time, regularly monitor liver function, and if abnormal timely inform the doctor to deal with.

The article "Related Factors of Cerebral Hemorrhage after Cerebral Infarction and the Effect of Atorvastatin Combined with Intensive Nursing Care" was retracted in 2023. Reasons: signs of a paper mill; compromised peer review; unreliable results or conclusions.

### 2.4. Indicator Evaluation

The differences in peripheral blood triglyceride (TG), total cholesterol (TC), high-density lipoprotein cholesterol (HDL-C), low-density lipoprotein cholesterol (LDL-C), National Institutes of Health Stroke Scale (NIHSS) score, and Glasgow Outcome Scale (GOS) score between the two groups were compared.

The following is the GOS score: 5 points: the neurological function of patients recovered well after treatment, and they could live normally; 4 points: patients with mild physical disability can participate in work under protection; 3 points: the degree of limb function disability of patients is relatively obvious, but they are aware of it and need special care in daily life; 2 points: patients in vegetative state; and 1 point: death of patients.

Before and after treatment, 5 mL venous blood samples were taken from two groups of patients under fasting state and centrifuged at 3000 r/min for 10 min after 1 h. Serum TC and other measurement indexes were detected by Hitachi 7600 automatic biochemical analyzer and supporting reagents.

National Institutes of Health Stroke Scale (NIHSS) mainly includes 11 items: level of consciousness, gaze, visual field, facial paralysis, upper limb movement, lower limb movement, limb ataxia, sensation, language, dysarthria, regression, and neglect. The total score is 0~42 points. The higher the score, the more serious the patient's neurological deficits: 0-1 point (normal), 1-4 points (mild), 5-15 points (moderate), 15-20 points (moderate to severe), and 21-42 points (severe).

### 2.5. Statistical Processing

In this study, the serum TC and other measurement indexes of patients were tested by normal distribution, which were in line with the approximate normal distribution or normal distribution, and expressed as $\bar{x}\pm s$. The *t* test was used for comparison between the two groups. *χ*^2^ test was used for comparison between groups of nongrade counting data; logistic regression method was used for the multivariate model; Mann-Whitney *U* test was used for comparative analysis between groups of grade counting data; using professional SPSS21.0 software for data processing, test level *α* = 0.05.

## 3. Results

### 3.1. Univariate Analysis Results of Basic Data

The basic data of the two groups were analyzed by single factor analysis. The age, NIHSS score at admission, proportion of patients with hypertension, and proportion of patients with atrial fibrillation in the observation group were higher than those in the control group (*P* < 0.05). TOAST classification and infarct size of observation group and control group were compared (*P* < 0.05, Table 1).

The article "Related Factors of Cerebral Hemorrhage after Cerebral Infarction and the Effect of Atorvastatin Combined with Intensive Nursing Care" was retracted in 2023. Reasons: signs of a paper mill; compromised peer review; unreliable results or conclusions.

### 3.2. Results of Multivariate Analysis

Logistic regression model was established with age, NIHSS score at admission, hypertension, atrial fibrillation, TOAST classification, and infarct size as independent variables. The results showed that higher score at admission, hypertension, atrial fibrillation, TOAST as small artery occlusion, and large infarct size were risk factors for hemorrhagic transformation in patients with cerebral infarction (*P* < 0.05, Table 2).

### 3.3. Comparison of Blood Lipid Levels between the Intervention Group and Conventional Group

Before treatment, the serum TC, TG, HDL-C, and LDL-C of the intervention group and the conventional group were not statistically different (*P* > 0.05). After treatment, the serum TC, TG, HDL-C, and LDL-C of the two groups were not statistically different as well (*P* > 0.05). The serum TC, TG, HDL-C, and LDL-C in both groups after treatment were significantly lower than those before treatment (*P* < 0.05, Table 3).

### 3.4. Comparison of NIHSS Scores between the Intervention Group and the Conventional Group

Pretreatment NIHSS score was compared between the two groups (*P* > 0.05). After two weeks and four weeks of treatment, the score was lower than that in the conventional group (*P* < 0.05, Table 4).

### 3.5. Comparison of Prognostic Outcomes between the Intervention Group and Conventional Group

The patients with GOS scores of 5 and 4 in the intervention group were 16.67% and 56.67%, respectively. The conventional group is 6.67% and 33.33%, respectively. The overall prognosis of the intervention group was better than that of the conventional group (*P* < 0.05, Table 5).

### 3.6. Imaging Data of Cases

Figure 1 shows a 63-year-old male patient with a history of hypertension for more than 10 years. Figures 1(a) and 1(b) are right basal ganglia lacunar infarction, Figures 1(c) and 1(d) are brainstem hemorrhage after thrombolysis, and Figures 1(e) and 1(f) are right thalamic hemorrhage breaking into ventricle.

## 4. Discussion

Cerebral hemorrhage transformation can lead to poor prognosis in patients with acute cerebral infarction, which is related to many factors such as inflammatory reaction of brain tissue around cerebral infarction, destruction of blood brain barrier, ischemia reperfusion injury, and opening of collateral circulation. Studies have found that the incidence of spontaneous hemorrhagic transformation is 3.8%-7.1% [11]. The coexistence of cerebral ischemia and cerebral hemorrhage lesions can cause the complication of the disease, and the anticoagulant, thrombolytic, and antiplatelet drugs cannot be used normally in the presence of cerebral hemorrhage, which cannot achieve the desired effect in the treatment of acute cerebral infarction. Therefore, active prevention and treatment should be given to cerebral hemorrhage transformation [12–15]. Statins are competitive inhibitors of 3-hydroxy-3-methylglutarate monoacylase A reductase, which can reduce the synthesis of cholesterol in the liver, increase the activity of low-density lipoprotein receptor on the surface of liver cells through feedback regulation, and accelerate the clearance of low-density lipoprotein. Statins have good effects in improving blood lipid metabolism and antiatherosclerotic plaque formation [16–19]. In addition, a large number of studies have confirmed that statins can improve endothelial cell function, reduce inflammation, stabilize plaque, and prevent thrombosis, which has a wide range of applications in the prevention and treatment of cardiovascular and cerebrovascular diseases [20–23].

The article "Related Factors of Cerebral Hemorrhage after Cerebral Infarction and the Effect of Atorvastatin Combined with Intensive Nursing Care" was retracted in 2023. Reasons: signs of a paper mill; compromised peer review; unreliable results or conclusions.

The results of logistic regression model showed that the increased NIHSS score at admission, hypertension, atrial fibrillation, TOAST classification of small artery occlusion, and large infarction lesions were the risk factors for hemorrhagic transformation in patients with cerebral infarction. Such patients should be given active prevention and treatment measures as high-risk groups in the future. Those with high NIHSS score at admission, TOAST classification of small artery occlusion, and large infarction lesions suggested severe neurological function, accompanied by obvious cerebral edema, which exerted great pressure on the injured cerebral vessels and increased the risk of bleeding transformation. Hypertension can lead to vascular endothelial injury, and vascular sclerosis is more serious; hypertension can also increase intracranial blood pressure, resulting in vascular rupture and cerebral hemorrhage. Atrial fibrillation is prone to thrombosis and increases the risk of cerebrovascular embolism, the degree of brain edema, and the risk of cerebral hemorrhage [24–26].

Early intensive nursing intervention can improve the prognosis of patients from the aspects of medication, diet, and complication prevention. The study found that early intensive care provided patients with low-salt and low-fat diet, but the effect of diet on blood lipid level was relatively small in a short period of time. In addition, both groups of patients took atorvastatin, which had obvious lipid-lowering effect and had relatively large effect on blood lipid level of patients. So the blood lipid levels of the two groups were similar [27–29].

The NIHSS score and GOS score were used to evaluate the condition and prognosis of patients. The results suggested that the use of atorvastatin calcium tablets combined with early intensive nursing intervention for patients with bleeding transformation was helpful to improve the prognosis of patients. This is because vascular stenosis and plaque instability are independent risk factors for cerebrovascular disease, and they are also important reasons for the increase of NIHSS. Atorvastatin alleviates cerebrovascular disease and improves prognosis by regulating lipid, anti-inflammatory, and antiatherosclerosis and maintaining plaque stability [30–32]. Early intensive nursing intervention reduced brain edema by raising the bed; using restraint belt prevented falling bed; timely help patients turn over, knock back, and massage compression site, reducing the risk of complications. Blood lipid elevation and blood flow retardation were prevented through diet guidance. Patients with rational drug use were monitored to ensure efficacy and reduce adverse reactions [33–35].

The article "Related Factors of Cerebral Hemorrhage after Cerebral Infarction and the Effect of Atorvastatin Combined with Intensive Nursing Care" was retracted in 2023. Reasons: signs of a paper mill; compromised peer review; unreliable results or conclusions.

Cerebral hemorrhage transformation is a common clinical complication. In this study, single factor analysis showed that hypertension, large infarction lesions, high NIHSS score at admission, atrial fibrillation, and small artery occlusion cerebral infarction could increase the risk of cerebral infarction complicated with hemorrhage transformation. This study also used atorvastatin calcium tablets combined with early intensive nursing intervention for patients and found that it was helpful to improve the prognosis of patients. In the future clinical work, statins should be used as one of the routine treatment of patients with cerebral infarction, and early intensive nursing intervention should be implemented in the treatment process to ensure curative effect and reduce adverse reactions.

In conclusion, hypertension, large infarction lesions, high NIHSS score at admission, atrial fibrillation, and small artery occlusion cerebral infarction can increase the risk of bleeding transformation in patients with cerebral infarction. For patients with bleeding transformation, atorvastatin calcium tablets combined with early intensive nursing intervention have certain value for improving the prognosis of patients.

## Figures and Tables

**Figure 1:** A 63-year-old male patient with a history of hypertension for more than 10 years. (a and b) Right basal ganglia lacunar infarction, (c and d) brainstem hemorrhage after thrombolysis, and (e and f) right thalamic hemorrhage breaking into ventricle.

**Table 1:** Univariate analysis results of basic data.

Index	Observation group (*n* = 60)	Control group (*n* = 90)	*t*/*χ*^2^	*P*
Age (years)	70.3 ± 5.2	68.2 ± 6.1	2.188	0.030
BMI (kg/m^2^)	25.1 ± 1.9	24.7 ± 2.2	1.151	0.252
NIHSS score (points)	13.29 ± 2.65	12.40 ± 2.38	2.144	0.034
GOS score (points)	9.45 ± 1.03	9.72 ± 1.16	-1.459	0.147
Time from onset to admission (h)	13.3 ± 2.4	12.6 ± 2.8	1.586	0.115
Male/female	37/23	46/44	1.623	0.203
Diabetes (%)	28 (46.67)	31 (34.44)	2.254	0.133
Hypertension (%)	41 (68.33)	45 (50.00)	4.946	0.026
Hyperlipidemia (%)	45 (75.00)	73 (81.11)	0.801	0.371
Coronary heart disease (%)	9 (15.00)	7 (7.78)	1.971	0.160
Atrial fibrillation (%)	13 (21.67)	6 (6.67)	7.322	0.007
Smoking (%)	25 (41.67)	31 (34.44)	0.803	0.370
Drinking (%)	29 (48.33)	36 (40.00)	1.018	0.313
TOAST type (%)			10.935	0.001
Atherosclerosis of large arteries	17 (28.33)	34 (37.78)		
Small artery occlusion type	33 (55.00)	26 (28.89)		
Other reasons	10 (16.67)	30 (33.33)		
Infarct size (%)			7.325	0.025
Large infarct	34 (56.67)	32 (35.56)		
Middle infarction	21 (35.00)	41 (45.56)		
Lacunar infarction	5 (8.33)	17 (18.89)		

The article "Related Factors of Cerebral Hemorrhage after Cerebral Infarction and the Effect of Atorvastatin Combined with Intensive Nursing Care" was retracted in 2023. Reasons: signs of a paper mill; compromised peer review; unreliable results or conclusions.

**Table 2:** Logistic regression model results.

Index	*β*	SE	Walds	*P*	OR	95% CI	
Age	0.611	0.443	1.902	0.201	1.842	0.773	4.390
NIHSS score	0.594	0.211	7.925	0.000	1.811	1.198	2.739
Hypertension (%)	0.701	0.335	4.379	0.046	2.016	1.045	3.887
Atrial fibrillation (%)	0.883	0.338	6.825	0.000	2.418	1.247	4.690
TOAST type	0.548	0.241	5.170	0.031	1.730	1.079	2.774
Infarct size	0.632	0.296	4.559	0.043	1.881	1.053	3.361
Constant term	1.627	0.740	4.834	0.040	5.089	1.193	21.702

**Table 3:** Comparison of blood lipid levels between the intervention group and conventional group $\bar{x}\pm s$.

Group	*n*	TC (mmol/L)		TG (mmol/L)	
		Before therapy	After treatment	Before therapy	After treatment
Intervention group	30	6.34 ± 0.68	4.70 ± 0.60^∗^	2.73 ± 0.50	1.84 ± 0.36^∗^
Control group	30	6.51 ± 0.72	4.84 ± 0.66^∗^	2.81 ± 0.46	1.89 ± 0.40^∗^
*t*		-0.940	-0.860	-0.645	-0.509
*P*		0.351	0.394	0.522	0.613

Group	*n*	HDL-C (mmol/L)		LDL-C (mmol/L)	
		Before therapy	After treatment	After treatment	Before therapy

Intervention group	30	0.90 ± 0.14	1.18 ± 0.18^∗^	3.85 ± 0.60	2.94 ± 0.47^∗^
Control group	30	0.88 ± 0.13	1.22 ± 0.20^∗^	3.97 ± 0.66	3.07 ± 0.51^∗^
*t*		0.573	-0.814	-0.737	-1.027
*P*		0.569	0.419	0.464	0.309

Note: compared with this group before treatment ^∗^*P* < 0.05.

**Table 4:** Comparison of NIHSS score between the intervention group and conventional group ($\bar{x}\pm s$, points).

Group	*n*	Before therapy	2 weeks after treatment	4 weeks after treatment
Intervention group	30	13.41 ± 2.61	8.43 ± 1.96^∗^	4.31 ± 1.10^∗^
Control group	30	13.17 ± 2.55	9.50 ± 2.11^∗^	5.20 ± 1.34^∗^
*t*		0.360	-2.035	-2.812
*P*		0.720	0.046	0.007

Note: compared with this group before treatment ^∗^*P* < 0.05.

**Table 5:** Comparison of prognostic outcomes between the intervention group and conventional group.

Group	*n*	5 points	4 points	3 points	2 points	1 point
Intervention group	30	5 (16.67)	17 (56.67)	5 (16.67)	2 (6.67)	1 (3.33)
Control group	30	2 (6.67)	10 (33.33)	8 (26.67)	7 (23.33)	3 (10.00)
*Z*		-2.238				
*P*		0.025				

The article "Related Factors of Cerebral Hemorrhage after Cerebral Infarction and the Effect of Atorvastatin Combined with Intensive Nursing Care" was retracted in 2023. Reasons: signs of a paper mill; compromised peer review; unreliable results or conclusions.

## Data Availability

No data were used to support this study.
